# Research Progress of Machine Learning and Deep Learning in Intelligent Diagnosis of the Coronary Atherosclerotic Heart Disease

**DOI:** 10.1155/2022/3016532

**Published:** 2022-04-26

**Authors:** Haoxuan Lu, Yudong Yao, Li Wang, Jianing Yan, Shuangshuang Tu, Yanqing Xie, Wenming He

**Affiliations:** ^1^The Affiliated Hospital of Medical School, Ningbo University, Ningbo 315020, China; ^2^Research Institute of Medical and Biological Engineering, Ningbo University, Ningbo 315211, China

## Abstract

The coronary atherosclerotic heart disease is a common cardiovascular disease with high morbidity, disability, and societal burden. Early, precise, and comprehensive diagnosis of the coronary atherosclerotic heart disease is of great significance. The rise of artificial intelligence technologies, represented by machine learning and deep learning, provides new methods to address the above issues. In recent years, artificial intelligence has achieved an extraordinary progress in multiple aspects of coronary atherosclerotic heart disease diagnosis, including the construction of intelligent diagnostic models based on artificial intelligence algorithms, applications of artificial intelligence algorithms in coronary angiography, coronary CT angiography, intravascular imaging, cardiac magnetic resonance, and functional parameters. This paper presents a comprehensive review of the technical background and current state of research on the application of artificial intelligence in the diagnosis of the coronary atherosclerotic heart disease and analyzes recent challenges and perspectives in this field.

## 1. Introduction

Coronary atherosclerotic heart disease (CAD) refers to a heart disease characterized by abnormal lipid metabolism, the accumulation of lipids and other substances in the blood in the coronary arteries, and the formation of atheromatous plaques. It can cause luminal narrowing or occlusion, leading to myocardial ischemia, oxygen deficiency, or necrosis, manifesting as chest pain, chest tightness, or myocardial infarction and other symptoms. Referred to as coronary heart disease (CHD), it is the most common type of atherosclerosis leading to organ lesions and a common disease that seriously endangers human health. Globally, in 2017, 126.5 million people lived with coronary heart disease, and 10.6 million new coronary heart disease cases occurred, resulting in 8.9 million deaths [1]. According to “Report on Cardiovascular Health and Diseases in China 2019: an Updated Summary,” the number of current CHD patients in China is about 11 million, and its incidence is rising significantly, corresponding to the fact that the mortality rate of also shows an obvious increasing trend, and in recent years, the mortality rate of coronary heart disease in rural areas has increased more significantly [2]. The accompanying problem is that the social health burden caused by coronary heart disease is also increasing. In the United States, CHD-related medical costs are expected to increase by 41%, from $126.2 billion in 2010 to $177.5 billion in 2040 [3]. CHD has become a serious public health problem worldwide.

Early detection, early diagnosis, and thus early intervention treatment are effective solutions to this problem. With the development of various auxiliary diagnostic techniques of coronary heart disease, it shows a diverse, precise, and individualized trend. In addition to the traditional gold standard (coronary angiography (CAG)) for CHD diagnosis [4], imaging techniques such as coronary CT angiography (CCTA) [5, 6], cardiac magnetic resonance, intravascular ultrasound (IVUS), and intravascular optical coherence imaging (IVOCT) [7] have been widely used for CHD diagnosis. With the further understanding of CHD, the luminal functional changes caused by coronary heart disease are becoming more appreciated by clinicians. Coronary functional parameters have been used as substantial medical evidence for guiding coronary revascularization strategies. Represented by fractional flow reserve (FFR) [8], it has been recommended by several international guidelines [9]. The imaging and functional tests described above have allowed the visualization of coronary stenosis, plaque burden, and myocardial ischemia quantitatively or qualitatively, which may not only diagnose coronary heart disease but also further guide the treatment strategies. However, patients diagnosed by the above methods often already have ischemic symptoms or severe coronary artery lesions. It is difficult to achieve early diagnosis. Besides, current diagnostic methods all have various limitations. For example, CAG, FFR, and intravascular imaging tests are all invasive procedures which have some risks and will obviously increase the financial burden on patients, making it difficult to truly generalize the above diagnostic methods, whereas relatively noninvasive CCTA is highly dependent on high-quality imaging results. Therefore, the existing techniques for CHD diagnosis still need to be further improved with the aim of diagnosing coronary heart disease early, noninvasively, and economically.

The advent of artificial intelligence (AI) has provided new ideas for improving CHD diagnostic techniques and has pioneered new areas of research. In recent years, the popularity of computer information systems and digital medical devices has caused the information capacity of hospital databases to expand continuously. These valuable medical information resources are very helpful in disease diagnosis and medical research. How to effectively utilize these data for intelligent diagnosis has become the focus of the attention of medical and informational researchers. The medical electronic data can be effectively integrated through AI algorithms, including the analysis and processing of the visualized imaging data, according to which the intelligent diagnostic model of coronary heart disease can be constructed, or the current imaging diagnostic methods can be improved. In addition, AI algorithms also have been applied to improve functional diagnosis of coronary heart disease, whereby convergence of imaging and functional diagnosis can be achieved. Overall, the current research of AI algorithms in the field of CHD diagnosis has been initially fruitful. In this paper, we will provide a review of recent applied studies of AI algorithms in CHD diagnosis and analyze the current challenges and perspectives in this field.

Due to the application of the existing AI algorithm in the research of CHD diagnosis has made some achievements, whether it is to construct intelligent diagnosis model or to improve imaging or functional methods, therefore, others have reviewed the related content [10–12]. Some reviewed the application of AI in the imaging diagnosis of coronary heart disease, while others reviewed the research progress of AI in the functional diagnosis of CHD. However, according to the author's investigation, there is no relevant review and the above content. On the basis of those reviews, this paper summarizes the AI research of intelligent diagnosis model, imaging, and functional diagnosis methods (see Figure 1).

The reminder of this paper is organized as follows: Section 2 briefly describes the AI algorithm, mainly about machine learning (ML) and deep learning (DL).  Section 3 introduces the application of AI in the field of coronary heart disease diagnosis.  Section 4 analyzes the existing problems in this field and makes some prospects for the future development.

## 2. AI

Artificial intelligence is a branch of computer science that aims to develop theory, methods, and application systems for modeling and expanding human brain intelligence. Artificial intelligence has unique advantages for the integration and processing of big data and has been widely applied in medical research. It can be expected that AI technology will play a more important role in the realization of precision medicine.

According to the different learning mechanisms, the learning methods of AI can be divided into machine learning and deep learning (see Figure 2). They have been widely used in medical research, which are introduced as follows.

### 2.1. ML

Machine learning is an important research area of AI, which refers to a range of techniques that solve complex big data problems by studying interactions. In the medical field, machine learning focuses on building automated clinical decision systems to help physicians make more accurate predictions compared to classical statistics [13]. More precisely, the distinction between ML and traditional statistics is not a methodological distinction, but a difference in purpose. The main focus of classical statistics is on inferring sample or population parameters, whereas machine learning focuses on algorithmically representing data structure and making predictions or classifications. Therefore, classical statistical and ML algorithms do not have clear boundaries but are often used to answer different questions.

Machine learning can be divided into supervised learning, unsupervised learning and reinforcement learning. Supervised learning obtains an optimal model by training labeled samples, then uses this model to map all the inputs to the corresponding outputs, and makes a simple judgment on the outputs to achieve classification. The sample data of unsupervised learning is not labeled, so it is usually necessary to cluster the data and select features by clustering. Reinforcement learning can be seen as a combination of supervised learning and unsupervised learning [14]. Specific machine learning algorithms include support vector machine (SVM), random forest (RF), decision tree (DT), genetic algorithm (GA), and Bayesian network (BN). These machine learning algorithms have been widely used in medical research and achieved good results.

### 2.2. DL

Deep learning is a new field in which AI algorithms have developed and burgeoned in recent years, which can be seen as an extension of machine learning. Deep learning establishes a mapping relationship from the underlying signal to the high-level semantics by building a hierarchical model structure that mimics the neural reflex circuits of the human brain, extracting features from the bottom to the top level of the input data step by step. This hierarchical model structure is called a neural network. Similar to ML algorithm, DL can also be divided into supervised learning, unsupervised learning, and reinforcement learning. Taking the convolutional neural network (CNN) algorithm as a representative, lots of medical studies have used the CNN algorithm [15], especially in the field of medical image processing. CNN algorithm shows clear advantages compared with machine learning algorithms. The image analysis process of machine learning involves several complicated steps, such as preprocessing of images, image segmentation, and selection of segments of interest, as well as statistical and machine learning algorithm classification. CNN algorithms can effectively simplify the process of image analysis and thus can help to save effort and improve work efficiency. There has been a significant increase in recent years in the application of CNN algorithms for quantitative analysis of medical imaging, such as the application of CNN algorithms to improve the detection rate of lung nodules [16], as well as the automated identification and classification of breast lesions [17, 18].

## 3. Application of AI in Diagnosis of CHD

As the most common cardiovascular disease, the diagnosis of coronary heart disease is highly dependent on visualized imaging data. The processing of imaging data is exactly the advantage of AI. Therefore, the interest of AI in the diagnosis of coronary heart disease is increasing year by year, and has achieved remarkable results.

Related research is mainly focused on intelligent diagnostic model and improvement of current imaging and functional diagnostic methods of coronary heart disease. The former is helpful in achieving an early diagnosis; the latter one makes relevant examination methods more convenient, precise, and diversified. The progress of machine learning algorithm and deep learning algorithm applied in CHD diagnosis will be described as follows.

### 3.1. Construction of an Intelligent Diagnostic Model for CHD Based on Medical Data

Data mining refers to the process of mining out useful information from complex data sets. It is possible to mine the data and discover the intrinsic associations of a large amount of data in a data set through AI algorithms. This mining for intrinsic connections does not exist with a clear hypothetical premise and can be regarded as an extension of traditional statistical methods. Traditional cardiovascular risk factors are helpful in the diagnosis of coronary heart disease. However, the diagnostic accuracy of these models constructed by statistical methods are limited accordingly. Compared with traditional statistical methods, AI methods are less demanding on the premise of data, not only can improve diagnostic accuracy, but also can discover some potential risk factors associated with the onset of coronary heart disease through data mining. So it has been applied to construct an intelligent aided diagnostic model of coronary heart disease in recent years.

#### 3.1.1. Intelligent Diagnosis Model of CHD Based on ML

Machine learning algorithm has been used to construct the intelligent diagnosis model of coronary heart disease. RF algorithm, DT algorithm, ensemble algorithm, and SVM algorithm are commonly used to build the model. They have good performance, ease of use and low computational burden, and are suitable for almost all CHD data sets. Kathleen et al. [19] developed an advanced integrated machine learning algorithm to apply adaptive Boosting algorithm to construct CHD intelligent diagnostic model. The developed integrated learning algorithm classification and diagnostic model was applied to 4 different diagnostic data sets. The results showed that 4 data corresponded to a model diagnostic accuracy of 80.14%, 89.12%, 77.78%, and 96.72%, respectively. Hassannataj et al. [20] constructed diagnostic models of coronary heart disease by four algorithms, respectively, in which a diagnostic accuracy of 90.50% was obtained by the diagnostic model constructed by RF algorithm. These studies reflect that the applications of machine learning algorithms have the potential to diagnose coronary heart disease through medical data from electronic medical record systems, which can help CHD diagnosis achieve earlier and more economical goals.

#### 3.1.2. Intelligent Diagnosis Model of CHD Based on DL

Although machine learning can mine and automatically learn the important feature information in the data set, so as to diagnose diseases efficiently, it is still unable to mine the temporal information of the data. Deep learning algorithms effectively compensates for the above deficiency. And compared with machine learning algorithms, deep learning algorithms can further improve diagnostic accuracy. Beunza et al. [21] compared the intrinsic validity and accuracy of neural network algorithms and several machine learning algorithms in diagnosing coronary heart disease. This study applied two software tools: R-Studio and Rapid Miner. When applying R-Studio software for analysis, the highest AUC was obtained for the diagnostic model constructed based on the neural network algorithm (AUC = 0.71). Compared with machine learning algorithm, the main disadvantage of neural network is that it takes more than 10 minutes to calculate. Recently, studies have proposed the application of the recurrent neural networks algorithm (RNN) to construct diagnostic models. In related tasks of temporal learning, CNN algorithms can only capture local feature information and need to assume that one piece of data is strictly in nature. Compared with that, RNN, such as long short-term memory neural network algorithm (LSTM), can capture useful information with different “Gates” and round the information without discarding so that the data with temporal information can be better processed [22]. Tan et al. [23] stack based convolutional LSTM algorithm to analyze ECG data from an open database of PhysioNet and constructed a CHD diagnostic model. It had a high diagnostic accuracy of 99.85%. In terms of running time, it took approximately 51 seconds to run a single epoch The above studies are sufficient to demonstrate that deep learning algorithms have good application prospects in the diagnostic field of coronary heart disease.  Table 1 shows the details.

### 3.2. AI Applied to CCTA

Coronary CT angiography has been widely used to evaluate patients with low to intermediate risk stable coronary heart disease because of its high sensitivity, specificity, and negative predictive value. Compared with coronary angiography, CCTA has the advantage of being able to diagnose coronary heart disease noninvasively and more economical. It is foreseeable that the clinical need for CCTA will expand even further in the future. However, CCTA is still not a substitute for coronary angiography in terms of positive predictive value in coronary heart disease. However, CCTA has high requirements for image quality. Low quality image data may cause deviation of results. Serious calcification and arrhythmia may also lead to image artifacts and affect the interpretation of results. At present, CCTA cannot replace coronary angiography in the positive predictive value of CHD. AI algorithm can improve the accuracy of CCTA in the diagnosis of coronary heart disease. The degree of coronary artery stenosis can be measured through automatic segmentation of CCTA images, and the potential information hidden in CCTA images can be mined, such as the type of plaque and coronary hemodynamic parameters.

#### 3.2.1. ML Applied to CCTA

Machine learning algorithms have been applied to image segmentation and automated measurement of CCTA images. Localizing the affected lesion segment and performing image segmentation are often seen as a preprocessing to detect coronary artery luminal stenosis. The detection of the severity of coronary artery stenosis is the most fundamental application of machine learning algorithm analysis on CCTA images. Current studies are relatively mature. Besides, identifying noncalcified plaques in CCTA images by machine learning algorithms and making classifications are also gradually carried out.

The detection of coronary stenosis by CCTA usually requires the reconstruction of a three-dimensional coronary tree. Automated extraction of the coronary tree by conventional CCTA may create bias and requires manual correction for use in clinical analysis. Machine learning algorithms can automatically identify biases resulting from reconstructing three-dimensional coronary trees, thus avoiding tedious manual modification. Cao et al. [24] performed refinements on the extracted reconstructed coronary tree automatically and iteratively based on DT, through 18 data sets to determine the optimal values of parameters involved in the model revision method and using 122 data sets for evaluation. It was shown that the proposed DT algorithm improved the accuracy of reconstructing the coronary tree compared with conventional coronary tree extraction methods. Machine learning algorithms can also automatically identify coronary obstructive lesions. Kang et al. [25]. applied SVM algorithms to detect lesions with coronary stenosis more than 25%. The sensitivity and specificity reached 93% and 95%, respectively. In addition, the detection of noncalcified plaques in CCTA has been a challenging issue due to the low density values of noncalcified plaques, which are usually similar to nearby blood and muscle tissues and difficult to identify. Machine learning algorithms can be helpful to identify noncalcified plaques in CCTA. Muhammad et al. [26] calculated the radial contour of noncalcified plaques by averaging image intensities in concentric rings around the vessel centerline. Then, it applied SVM algorithms to identify coronary lesion segments. Plaque localization accuracy was calculated using the dice similarity coefficient (DSC) and achieved an average DSC of 83.2%. Therefore, machine learning method can be used to process CCTA image processing and improve the accuracy of diagnosis of coronary heart disease and has good application value.

#### 3.2.2. DL Applied to CCTA

The advantage of deep learning algorithms over machine learning is that it further simplifies the steps of image analysis and improves the automation of image analysis. Zreik et al. [27] achieved the integration of classifying coronary plaque types and detecting the severity of coronary stenosis by multitasking a recursive CNN algorithm. The proposed method achieved an accuracy of 0.77. Deep learning algorithms can also be used to analyze coronary blood flow and calculate coronary functional parameters. Fractional flow reserve calculation based on CCTA images is a representative study. Kumamaru et al. [28] designed a fully automated three-dimensional deep learning model to input CCTA image data and automatically analyze calculated fractional flow reserve without manual input. The model consists of a series of DL algorithms: a condition generating adversarial network algorithm, a three-dimensional convolutional trapezoidal network algorithm, and two independent neural network integrated virtual adversarial training algorithms. The Monte Carlo Cross-Validation showed that the deep learning algorithm achieve an AUC of 0.78.

In the application of reconstruction of coronary artery trees, deep learning algorithms improve the automation of reconstruction of coronary artery trees in addition to their accuracy [29]. But whether machine learning algorithms or deep learning algorithms, the process of reconstructing coronary trees is complex which increases the difficulty of image processing and the burden of computational analysis. Therefore, some scholars have proposed the reconstruction of coronary tree with left ventricular myocardial replacement by deep learning algorithm for the diagnosis of patients with functional coronary stenosis. Zreik et al. [30] used multiscale CNN algorithm to segment left ventricular myocardium. Subsequently, the algorithm encoded it using an unsupervised convolutional autoencoder and then classified it using SVM algorithm based on extracted features. The results were evaluated by 50 times 10-fold cross-validation and showed the combined algorithm model obtained an AUC of 0.74 ± 0.02. A retrospective study conducted by Hamersvelt et al. [31], in which the CNN algorithm was used, analyzed left ventricular myocardial images in 136 patients who underwent CCTA within 1 year prior to interventional fractional flow reserve. Aiming at the diagnosis of patients with significant functional stenosis, the result showed that the proposed method improved a diagnostic performance (AUC = 0.76) compared to the classification based on coronary stenosis alone (AUC = 0.68).

To summarize, Table 2 lists representative ML and DL application examples in CCTA.

### 3.3. AI Applied to CAG

Coronary angiography is the gold standard of clinical diagnosis of coronary heart disease, which can directly show the location, severity, characteristics, and collateral circulation status of coronary obstructive lesions. Current clinical efforts to interpret coronary angiographic findings primarily involve the experience of the operator with visual inspection or quantitative coronary angiography (QCA). Visual inspection is the more commonly used clinical interpretation method, which requires the operator to have certain experience in image interpretation, and it is more subjective. QCA allows for computer-based analysis of contrast images and quantification of stenosis, length, and minimum lumen diameter, with relatively objective results. The limitation lies in the lack of accuracy in the case of diffuse lesions and vascular distortion [32]. AI algorithms can assist in the analysis of coronary angiographic findings, both objectivity and automation are considered. However, current coronary angiography cannot clarify whether a coronary artery stenosis is a functional stenosis. But coronary angiographic images may contain potential information for diagnosing functional stenosis. AI algorithms can extract this potential information and make a diagnosis of functional stenosis.

#### 3.3.1. ML Applied to CAG

Coronary angiography can only provide coronary anatomically relevant parameters, and it is difficult to integrate coronary anatomic and functional parameters. A major reason for the incomplete matching between the severity of coronary stenosis and myocardial ischemia lies in the fact that myocardial ischemia is determined by multiple factors. And the accuracy of fractional flow reserve, a functional parameter, is less than 70% when diagnosed based solely on the degree of stenosis revealed by coronary angiography [33]. Machine learning algorithms can mine additional information in contrast images to improve the accuracy of diagnosing fractional flow reserve. Cho et al. [34] used the XG Boost algorithm for feature extraction from the angiographic results of 1501 patients with coronary artery lesions. Scattering search selected 12 high-level features and constructed a classification model using these 12 features for fractional flow reserve. The results showed that the sensitivity, specificity, and accuracy of the model were 84%, 80%, and 82% (AUC = 0.87). The accuracy of external verification was 85% (AUC = 0.87), which improved the classification accuracy compared with a classification model based on the severity of coronary stenosis alone.

#### 3.3.2. DL Applied to CAG

Automated segmentation of the coronary arteries is currently difficult to achieve with either 2D or 3D quantitative coronary angiography. Although computer-aided tools such as edge detection are used, manual correction is still necessary for accurate segmentation of coronary artery. Deep learning algorithm effectively solves the training problem of quantitative coronary angiography. Yang et al. [35] proposed a robust method for large vessel segmentation using deep learning model of full CNN algorithm. On examining the contrast images of 3302 diseased vessels from 2042 patients, the deep learning network accurately identified and segmented the major vessels in coronary angiography. The results showed that the average F1 score of the algorithm reached 0.917 and 93.7% of the images had F1 scores more than 0.8. The narrowest region of the stenosis can be clearly visualized with a high degree of continuity. This method validated the robustness and predictability of external data sets with different image features. By applying deep learning algorithm segmentation, QCA analysis can be further automated, thus facilitating the application of QCA based interpretation image technology.

### 3.4. Application of AI in Intravascular Imaging

Intravascular imaging techniques (including IVUS and IVOCT) have been proved to have advantages in assessing plaque progression or regression, identifying vulnerable plaque, assessing plaque burden, and guiding interventional therapy. The clinical uses of IVUS and IVOCT have further advanced the understanding of the pathophysiology of coronary heart disease among clinical workers. These two technologies have their own advantages and disadvantages. As IVUS enables precise description of plaque structure, it lacks spatial resolution, while IVOCT enables high-resolution measurement of the fibrous cap but has limited ability to penetrate the arterial wall. AI algorithm can automatically segment and process the plaque images obtained by IVUS and IVOCT, so as to obtain the plaque information accurately, quickly, and objectively and make up for their respective defects to a certain extent.

#### 3.4.1. ML Applied to IVUS

IVUS is a medical imaging technique that combines ultrasound technology and catheter technology. It can be used to examine the inner walls of blood vessels by using a special catheter with an ultrasound probe attached to the end. The high sensitivity of IVUS in detecting atherosclerosis, identifying plaque types, and quantifying atheroma burden have been widely recognized by clinical workers.

IVUS can be used to identify the coronary artery lumen and adventitia. However, the presence of high noise, artifacts, and anatomical structures (e.g., bifurcations, calcifications, and fibrotic plaques) often impedes proper segmentation of the vessel wall. Machine learning can improve segmentation efficiency. Lucas et al. [36] used SVM algorithm to automatically detect luminal, media, adventitia, and perivascular tissues. Different image structures were detected by RF algorithm, and the classification is modified according to the detected structures. The resulting classification maps were then fed into a segmentation method based on deformable contours to detect the lumen intima and media adventitia interfaces. The Jaccard measure of the proposed automatic segmentation method is 0.88 ± 0.08.

IVUS is also helpful for the detection of vulnerable plaques. However, the progression of plaques cannot be analyzed. Machine learning algorithms can achieve the prediction of the progression of vulnerable plaques, which is significant for the prognosis evaluation of patients. Wang et al. [37] established a fluid structure interaction model based on the IVUS coronary plaque data of 9 patients. Plaque vulnerability index was used to measure plaque vulnerability. Generalized linear mixed regression model, SVM, and RF algorithm were used to predict plaque vulnerability. The results showed that RF algorithm had the highest prediction accuracy (91.47%), and it is 5.91% higher than the generalized linear mixed regression model.

#### 3.4.2. DL Applied to IVUS

Deep learning algorithms further improve the efficiency of image segmentation based on machine learning algorithms. CNN has achieved significant improvements in automatic patch segmentation. Jun et al. [38] used four AI algorithm classifiers (including FNN, KNN, RF, and CNN algorithms) to classify IVUS images. The results show that CNN algorithm obtains the best AUC (AUC = 0.911). Yang et al. [39] proposed a deep structure based on complete convolution network algorithm, called the DPU-Net, which is used for automatic segmentation of lumen and outer membrane of IVUS image. Its segmentation performance is better than other existing methods.

Deep learning algorithm also helps to integrate the coronary plaque parameters provided by IVUS with the functional parameters, which will be of great significance for interventional physicians to make treatment decisions. The examination methods to obtain coronary plaque parameters or functional parameters in current clinical practice are both complex and time-consuming, and therefore guidance of treatment decisions is usually made based on only one of these examinations. The availability of simultaneous access to both parameters would be more instructive for the development of treatment options. Lee et al. [40] randomly divided 1328 patients with non-left main coronary artery lesions into training set and test set according to the ratio of 4 : 1. The IVUS image was segmented automatically by the CNN algorithm. 99 IVUS features and 6 clinical variables (age, gender, body surface area, vascular type, involved segments, and lesions of proximal left anterior descending branch) were used for training and 5-fold cross-validation. Non-overlapping test samples were used to evaluate the diagnostic performance of binary classifiers (L2 penalty logistic regression, ANN, RF, AdaBoost algorithm, CatBoost algorithm, and SVM) for detecting ischemic lesions. The results showed that when the lesions in the test set were classified as lesions with FFR ≤ 0.80 and FFR > 0.80, the overall diagnostic accuracy of predicting FFR ≤ 0.80 was 82%.

#### 3.4.3. ML Applied to IVOCT

IVOCT is similar to IVUS, but optical pulse and optical technology are used for the visualization of coronary artery. The resolution is higher than IVUS, which can detect vulnerable plaque, stent intimal hyperplasia and stent wall sticking, etc,, while the penetration is less than IVUS. At present, the analysis of IVOCT image is still limited to the manual process of clinicians. It is often difficult to get different evaluation results due to the subjective differences observed by different doctors. Machine learning algorithm can be used to analyze IVOCT images to make up for this problem. The automatic classification of calcified plaque, fibrosis plaque, and lipid pool can be realized by using machine learning algorithm to segment IVOCT images. Kolluru et al. [41] developed a machine learning algorithm to classify the voxel plaque types in IVOCT images automatically. To train and test the classifier, 300 images were used, and each voxel was labeled fibrosis, lipid rich, calcification, or other. The algorithm automatically extracted the light attenuation, light intensity, and texture features of each voxel to build a multiclass DT algorithm classifier. The cross-validated results showed that 96% ± 0.01%, 90% ± 0.02%, and 90% ± 0.01% classification accuracies were achieved for fibrotic, lipid rich, and calcified plaques, respectively.

#### 3.4.4. DL Applied to IVOCT

Deep learning algorithm improves the automation of patch segmentation and realizes the automatic segmentation of patches [42]. Lee et al. [43] developed a full-automatic semantic segmentation model of plaque in IVOCT image based on CNN algorithm. It realized the high sensitivity and high specificity classification of lipid and calcified plaque (sensitivity and specificity are 87.4%/89.5% and 85.1%/94.2%, respectively). Xu et al. use four deep CNN algorithms: AlexNet algorithm, GoogleNet algorithm, VGG-16 algorithm, and VGG-19 algorithm to extract the depth characteristics of atheroma. These features are evaluated by a data set containing 360 IVOCT images. Data enhancement is applied to each classification scheme training set. Linear SVM algorithm classifies normal IVOCT image and IVOCT image and fibroatheroma. The results show that the depth of the fibroatheroma can be extracted in the classification of the fibroatheroma with high accuracy [44].

In Table 3, we summarized the applications of AI in intravascular imaging.

### 3.5. AI Applied to Cardiac MRI

Magnetic resonance imaging was first used in the detection of nervous system diseases such as cerebral infarction and cerebral ischemia. With the improvement of the performance of MRI equipment and the progress of hardware and software technology, it has gradually been used to examine cardiovascular diseases. The MRI can be used to show the structure, function, perfusion, activity, and extent of myocardial infarction in patients with coronary heart disease. The research of AI algorithm applied to cardiac MRI is also increased gradually. The related research mainly focused on the application of AI algorithm to the image processing of cardiac MRI, including reducing image acquisition and reconstruction times, increasing spatiotemporal resolution, and the analysis of myocardial blood perfusion However, because cardiac magnetic resonance is more used in the diagnosis and analysis of cardiomyopathy than in the diagnosis or evaluation of coronary heart disease in practical clinical application, the research of artificial intelligence algorithm in the diagnosis of coronary heart disease by magnetic resonance is also less carried out.

#### 3.5.1. ML Applied to Cardiac MRI

The acquisition of MRI images usually requires the subjects to keep quiet for a period of time. The body movement or breathing movement of the patient may produce image artifacts such as ghosting, blurring, and smearing, thus reducing the image quality and its diagnostic value. Machine learning algorithm can automatically identify the motion artifacts of MRI images, thus eliminating the artifact interference and improving the accuracy of diagnosis. Motion is simulated by Cartesian sampling and shows how the effect of motion manifests in ghosts and blurry images. In addition, with radial acquisition, image structures can be made clearer and show robustness to small motion inconsistencies. Benedikt et al. [45] supervised learning methods based on stochastic decision forest algorithm detect motion artifacts in the reconstruction of MRI. According to the motion trajectory, three common spatial sampling modes are used: Descartes, radial, and spiral. The results show that the ML algorithm can learn the characteristics of motion artifact very well and improve the recognition rate of motion artifact. The classification accuracy for texture features increased from 77.1% for the lowest level of artefacts to 91.8% for the highest level.

#### 3.5.2. DL Applied to Cardiac MRI

In the image postprocessing of cardiac MRI, deep learning algorithm shows the advantages of simplification, high automation, and hidden information extraction. The automatic segmentation and rearrangement of myocardial tissue by CNN algorithm for the automatic identification of infarcted myocardial tissue by features such as image texture is of great significance for patients with myocardial infarction. Baessler et al. [46] applied deep learning algorithm to analyze the texture of cardiac MRI, which selected the features of the texture based on the reproducibility and correlation analysis to distinguish the myocardial infarction tissue from the normal tissue. The AUC displayed under the multiple logic regression analysis was 0.92, which indicated that the deep learning algorithm can better distinguish the myocardial tissue and the infarction tissue.

### 3.6. Application of AI in Functional Diagnosis of CHD

Functional diagnosis of coronary heart disease has become the most important basis for guiding revascularization strategies on the basis of coronary imaging. It plays a key role in the characterization of critical lesions, the identification of target lesions in multivessel disease, and single vessel diffuse disease. At present, functional parameters of coronary heart disease commonly used in clinical practice include FFR, coronary CT angiography derived fractional flow reserve (CT-FFR), quantitative flow ratio (QFR), intravascular ultrasound derived fractional flow reserve (UFR), and optical coherence imaging derived fractional flow reserve (OFR), among which FFR is the gold standard of coronary artery functional parameters. CT-FFR, QFR, UFR, and OFR are derived from coronary imaging evaluation, which take into account the dual information of anatomy and function. These parameters are in the rising phase of clinical research and application.

FFR is the most classic functional evaluation parameter. It represents the ratio of the maximum blood flow of the myocardium in the distal area of the coronary artery stenosis to the maximum blood flow of the myocardium in the area of the coronary artery without stenosis. The value can be approximately the ratio of the mean pressure (PD) in the distal area of the lesion to the mean pressure (PA) in the proximal area (FFR ≈ Pd/PA). A prospective study showed that when FFR ≤ 0.80, it indicates that the stenosis needs revascularization, while FFR > 0.80 delayed intervention benefits more [47]. FAME and FAME-II studies confirmed that FFR-guided percutaneous coronary intervention patients had better prognosis than coronary angiography [47, 48].

CT-FFR is a noninvasive functional parameter based on coronary CT angiography, which has the advantages of noninvasive and rapid diagnosis. DISCOVER-FLOW and DeFACTO studies have confirmed that CT-FFR can accurately diagnose and exclude coronary artery functional stenosis [49, 50]. The core principle of CT-FFR is computational fluid dynamics (CFD). Coronary arteries in maximal hyperemia were simulated by CCTA images in the resting state, and three-dimensional coronary trees were reconstructed. Coronary flow was simulated as Newtonian fluid by Navier Stokes equation. CT-FFR was finally calculated by computer integrated simulated coronary arteries with blood flow parameters.

QFR is another noninvasive functional parameter based on the three-dimensional reconstruction image of coronary angiography and the principle of hydrodynamics. The principle is that at the end of diastole of the cardiac cycle, the angiographic images with the difference of two angles greater than 25° and the velocity of 15 frames per second are collected, and the three-dimensional reconstruction of the coronary artery is carried out. If the automatically reconstructed lumen contour does not conform to the real lumen boundary, it is necessary to manually sketch and proofread and select the starting and ending points of blood vessels. The system automatically selects the contrast flow image and calculates the contrast flow time, velocity, and average volume flow by TIMI frame counting method. The virtual pressure withdrawal curve of quantitative blood flow fraction was reconstructed, and the relevant parameters of the lesion site were calculated to obtain QFR [51].

CT-FFR and QFR are essentially functional parameters obtained by applying AI algorithm to image postprocessing (CCTA and CAG). The potential hemodynamic features in CCTA or coronary angiography images can be mined by using AI algorithm, and the functional parameters can be obtained. However, the accuracy of CT-FFR and QFR still needs to be further improved. Research shows that optimizing AI algorithm and extracting more image features can help to improve the accuracy of CT-FFR and QFR [49]. In addition, intelligent analysis of intracoronary imaging (IVUS and IVOCT) to obtain FFR has become the focus of research.

In addition to the above parameters, the microvascular resistance (IMR) is used to evaluate the function of coronary microcirculation. The coronary flow reserve (CFR) is used to evaluate the function of the whole coronary circulation, including epicardial vessels and microcirculation. There are few researches on the application of AI algorithm in IMR and CFR, which is related to the relatively fewer clinical application of both.

#### 3.6.1. ML Applied to Functional Diagnosis of CHD

The application of machine learning algorithm in functional diagnosis of CHD mainly focuses on CT-FFR. The original method to obtain CT-FFR is to use computational fluid dynamics to postprocess CCTA results and then calculate CT-FFR. CT-FFR based on computational fluid dynamics calculation has been proved to have good correlation with FFR of invasive measurement and improve the diagnostic efficiency of CCTA [49, 50, 52–54]. Its major limitation is that it puts forward higher requirements for the performance of the computer and needs to take into account the problem of computing time. Machine learning algorithm can effectively simplify the image postprocessing program of CCTA. Coenen et al. [55] enrolled 351 patients who received both CCTA and FFR from five heart centers in Europe, Asia, and the United States and measured the FFR of 525 coronary arteries. In this study, machine learning algorithm and computational fluid dynamics were used to post process CCTA images, and CT-FFR was calculated. FFR was used as the gold standard to evaluate their diagnostic efficiency. The results show that CT-FFR based on machine learning algorithm can correctly classify stenotic lesions and its efficiency is equivalent to that of CT-FFR based on computational fluid dynamics. The former also effectively simplifies the calculation program.

CT-FFR based on machine learning algorithm can also help to predict major adverse cardiac events (MACE). Doeberitz et al. [56] retrospectively analyzed the data of 82 patients who received CCTA and coronary angiography at the same time and followed up the incidence of MACE. In this study, ML algorithm was used to quantify semiautomatic plaques of lesions causing MACE and the lesions in the control group. The predictive value of combined plaque markers and CT-FFR for MACE was evaluated. The results showed that the plaque markers extracted by CCTA and CT-FFR based on machine learning algorithm had higher predictive value for MACE compared with the stenosis classification determined only by CCTA.

Therefore, the application of machine learning algorithm in CT-FFR not only improves the diagnosis efficiency, effectively simplifies the calculation program, and saves the calculation time, but also has higher value for the prediction of MACE.

#### 3.6.2. DL Applied to Functional Diagnosis of CHD

Deep learning algorithm has more advantages in image segmentation compared with machine learning algorithm, and it has been widely used in noninvasive functional diagnosis. In recent years, DL algorithms have been applied to the research of CT-FFR, QFR, UFR, and OFR.

CT-FFR based on deep learning algorithm can also simplify the calculation procedure, reduce the calculation time, and help to evaluate the prognosis of patients [57, 58]. Based on deep learning algorithm (multilayer neural network algorithm), Kishi et al. [59] extracted the anatomic features of coronary arteries reconstructed by CCTA and constructed a computed model of CT-FFR that conformed to the rules of computational fluid dynamics. The operator was able to automatically analyze and calculate FFR from the model by only entering information such as vessel diameter and branch vessel length in the coronary tree reconstructed by CCTA. Compared with the original CT-FFR calculation, the calculation speed of the model is increased by about 80 times, and the calculation time is reduced to 2.4 seconds. In order to improve the accuracy of CT-FFR, the plaque features and hemodynamic features in CCTA images can be extracted by using deep learning algorithm, and CT-FFR can be calculated comprehensively. Doeperitz et al. [60] analyzed 84 patients who measured FFR after CCTA examination. The plaque and hemodynamic features in CCTA images were extracted by deep learning algorithm, and CT-FFR was calculated. Compared with CT-FFR, which only extracts hemodynamic characteristics, this method shows higher accuracy.

Although CT-FFR based on deep learning algorithm shows many advantages, there are still some limitations: (1) The computer-simulated coronary artery cannot fully simulate the real coronary artery, and there are differences in the elasticity of different patients. Whether the model reconstructed by deep learning algorithm can reflect the elasticity of coronary artery is still to be explored. (2) Currently, CT-FFR–related clinical research does not include patients who have had myocardial infarction or have received revascularization. (3) Compared with FFR, the results of CT-FFR generally underestimated the degree of lesions. In the future, further research on CT-FFR can be carried out in view of these limitations.

Different from CT-FFR, QFR is calculated by using deep learning algorithm on the basis of coronary angiography. Its accuracy is higher, and it can directly guide the treatment strategy of coronary heart disease after coronary angiography. At present, several multicenter and prospective clinical studies related to QFR have been carried out. The completed research on FALVOR study, FALVOR II China, FALVOR II Europe Japan, and WIFI II have fully proved the effectiveness of QFR and its good correlation with FFR [33, 51, 61, 62]. The ongoing FALVOR III China study is expected to answer the correlation between QFR and the clinical prognosis of patients [63]. Compared with traditional FFR, QFR is a noninvasive functional index which is more convenient and economical to obtain and can directly guide the intervention strategy after coronary angiography in the catheter room. It is expected to be the mainstream approach for evaluating the functional stenosis of the catheter.

FFR based on intravascular imaging results is a breakthrough in the application of deep learning algorithm in the diagnosis of coronary artery function. The representative research results include UFR and OFR based on deep learning algorithm. The original UFR and OFR are calculated based on computational fluid dynamics algorithm [64, 65]. The replacement of the computational fluid dynamics algorithm with deep learning algorithms effectively improves the utilization of imaging data. It extracts more image features to calculate FFR and reduces computational time. Yu et al. conducted a study to analyze the correlation between UFR and FFR based on deep learning algorithm. The UFR and FFR of 167 coronary artery lesions in 94 patients were compared. The results showed that the accuracy, sensitivity, specificity, positive predictive value, negative predictive value, positive likelihood ratio, and negative likelihood ratio of UFR diagnosis FFR ≤ 0.80 were 92%, 91%, 96%, 96%, 91%, 25.0, and 0.10, respectively. It is proved that UFR based on deep learning has a strong correlation and consistency with FFR. Furthermore, UFR based on deep learning has fast computing time and good analysis reproducibility [66]. In the aspect of OFR research, scholars such as Tu and others analyzed the correlation between OFR and FFR based on deep learning algorithm. The results show that OFR based on deep learning algorithm has reached 90.5% of accuracy [67]. Based on the image of intravascular imaging, FFR obtained by deep learning algorithm cannot only integrate the parameters of coronary plaque and functional parameters, but also help to predict the occurrence of adverse events in patients, which is of great clinical significance.

## 4. Challenges and Prospects

Traditional methods of coronary heart disease diagnosis can be divided into two aspects: imaging diagnosis and functional diagnosis. Imaging diagnosis methods mainly include CCTA, CAG, and intracavitary imaging (IVUS, IVOCT). Functional diagnosis methods mainly refer to FFR, IMR, and CFR. In clinical practice, traditional diagnosis methods can only obtain single diagnosis information. For example, coronary angiography can only obtain the information of coronary artery anatomy, but not the information of plaque and hemodynamic changes. IVUS or IVOCT can analyze coronary plaque, but it cannot obtain hemodynamic parameters of the vessels and cannot evaluate the severity of myocardial ischemia correctly. How to obtain the anatomical or functional information through one method and guide the treatment strategy of coronary heart disease more accurately is an important research direction for improving the diagnosis method of CHD.

In this paper, we describe the progress of machine learning and deep learning algorithms for CHD diagnosis (see a summary in Table 4), including the construction of intelligent diagnostic models for coronary heart disease and the applications of AI in the imaging and functional diagnostic methods. In addition, the simultaneous acquisition of coronary imaging and functional information using AI technology is also a research hotspot. Diagnostic methods such as CT-FFR, QFR, UFR, and OFR have emerged.

The intelligent diagnosis models of coronary heart disease cannot completely replace the traditional method to confirm the diagnosis of CHD at this time. It can only be used for early screening of CHD or noninvasively assisted diagnosis. Its accuracy still needs to be further improved. The main reason for this is that currently established clinical databases for coronary heart disease are not uniform standards and of mixed quality. The constructed models have limited diagnostic efficacy and lack sufficient validation with big data. Therefore, the construction of a standardized and large sample coronary heart disease medical database will be an important direction of future research, which will help to construct a higher quality diagnostic model.

The selection of AI algorithm is another important factor to determine the effectiveness of intelligent diagnosis method. The existing research has proved that the deep learning algorithm may have more advantages in the accuracy and speed of calculation especially in the processing of medical image. Therefore, further optimization of deep learning algorithms, such as CNN, AlexNet, and RNN, will also be an important research direction to improve the level of intelligent diagnosis of coronary heart disease, which deserves attention.

In terms of coronary functional diagnosis, some original works have been carried out in China such as the development of tools such as QFR, UFR, and OFR. They have gradually been promoted and applied in clinical applications. Most of the current studies were limited to the correlation between the abovementioned derived FFR and classic FFR. Further validation of its correlation with clinical prognostic outcomes is needed. At the same time, studies using AI to directly determine myocardial perfusion function have also been conducted. Betancur et al. [68] trained and analyzed raw quantitative perfusion polar maps from myocardial single photon emission computed tomography (SPECT) by deep learning algorithms and constructed a coronary heart disease prediction model. The results show that the accuracy of the model based on deep learning in predicting coronary heart disease is higher than that of the current clinical method. It shows another research direction to use AI technology to mine myocardial perfusion information in SPECT and coronary CT angiography to determine the severity of myocardial ischemia directly.

Although AI algorithms show many advantages in CHD diagnosis, the current problems and challenges remain. Firstly, the construction of a CHD diagnostic model relies on the establishment of data sets, the quality of which can directly affect the accuracy of the diagnostic model. Secondly, AI algorithms suffer from insufficient interpretability, akin to a “black box.” It can discover but fail to account for an intrinsic link between data sets that is often involved in pathophysiological disease mechanisms that currently cannot be directly explained by AI algorithms. The efficacy of AI algorithms needs further enhancement, as well as stability and interpretability. How to unify research that is currently refuted and form industry standards with relevant guidelines will also be a focus of future work.

In summary, the application of AI algorithms in the intelligent diagnosis of coronary heart disease has many advantages, contributing to the realization of an early, noninvasive, precise, and economical diagnosis of coronary heart disease. In the future, with the establishment of medical big data centers and continuous optimization of AI algorithms, the intelligent assisted diagnosis method of coronary heart disease will surely be more stable and accurate, with promising applications.

## Figures and Tables

**Figure 1:** Current status of AI applied in CHD diagnosis.

**Figure 2:** Relationship of AI,ML, and DL.

**Table 1:** AI applications in intelligent diagnosis model.

Method	Variable	Data	Measure	Value	Calculate time or cost	Paper
ML	29	303; 294; 200; 123	Accuracy	80.14% 89.12% 77.78% 96.72%	—	[19]
	55	303	Accuracy	90.50%	—	[20]
DL	16	4240	AUC	0.71	More than 10 minutes	[21]
	ECG signals	38120	Accuracy	99.85%	Approximately 51 seconds to run a single epoch	[23]

**Table 2:** AI applications in CCTA.

Method	Tasks	Data	Measure	Value	Calculate time or cost	Paper
ML	Modifications to the reconstructed coronary tree	122	Average quality score	93 ± 4	Within 2 minutes	[24]
	Identification of the degree of coronary stenosis	42	AUC	0.94	Less than 1 second	[25]
	Characterization of coronary plaques	32	DSC	83.2%	—	[26]
DL	Coronary plaque characterization and detection of coronary stenosis	163	Accuracy	77%	—	[27]
	Calculation of coronary functional parameters	1052	AUC	0.78	A few seconds	[28]
	Segmentation of left ventricular myocardium and calculation of coronary functional parameters	126	AUC	0.74 ± 0.02	—	[30]
	Segmentation of left ventricular myocardium and calculation of coronary functional parameters	126	AUC	0.76	—	[31]

**Table 3:** AI applications in intravascular imaging.

Application	Method	Tasks	Data	Measure	Value	Calculate time or cost	Paper
IVUS	ML	Lumen image segmentation	435	Jaccard measure	0.88 ± 0.08	—	[36]
		Prediction of progression to vulnerable plaque	748	Accuracy	91.47%	—	[37]
	DL	Plaque image segmentation	12325	AUC	0.911	3,584 CUDA cores and 12GB of GPU memory	[38]
		Lumen image segmentation	435	Jaccard measure	0.869	Run in 0.03 seconds	[39]
		Extraction of coronary plaque parameters and prediction of functional parameters	1328	AUC	0.84-0.87	—	[40]
IVOCT	ML	Plaque image segmentation and composition classification	300	Accuracy	96% ± 0.01% 90% ± 0.02% 90% ± 0.01%	Under 4 seconds when run on a standard 12-core CPU	[41]
	DL	Fully automated semantic segmentation of plaques	4892	Sensitivity/specificity	87.4%/89.5%; 85.1%/94.2%	0.27 seconds of each image	[43]
		Feature extraction and classification of fibroatheromas	360	Accuracy	76.39%	—	[44]

**Table 4:** A summary of AI applications in CHD.

Fields	Paper	Algorithm	Measure	Value	Calculate time or cost
Intelligent diagnosis model	Kathleen et al. [19]	Adaptive boosting algorithm	Accuracy	96.72%	—
	Hassannataj et al. [20]	RF	Accuracy	90.50%	—
	Beunza et al. [21]	CNN	AUC	0.71	More than 10 minutes
	Tan et al. [23]	LSTM	Accuracy	99.85%	Approximately 51 s to run a single epoch
CCTA	Cao et al. [24]	DT	Average quality score	93 ± 4	Within 2 minutes
	Kang et al. [25]	SVM	AUC	0.94	Less than 1 second
	Muhammad et al. [26]	SVM	DSC	83.2%	—
	Zreik et al. [27]	CNN	Accuracy	77%	—
	Kumamaru et al. [28]	DL	AUC	0.78	A few seconds
	Zreik et al. [30]	CNN SVM	AUC	0.74 ± 0.02	—
	Hamersvelt et al. [31]	CNN	AUC	0.76	—
CAG	Cho et al. [34]	XG boost	AUC	0.87	—
	Yang et al. [35]	CNN	F1	0.917	36236 seconds of training time
IVUS	Lucas et al. [36]	SVM RF	Jaccard measure	0.88 ± 0.08	—
	Wang et al. [37]	RF	Accuracy	91.47%	—
	Jun et al. [38]	CNN	AUC	0.911	3,584 CUDA cores and 12GB of GPU memory
	Yang et al. [39]	DPU-net	Jaccard measure	0.869	Run in 0.03 seconds
	Lee et al. [40]	CNN	AUC	0.84-0.87	—
IVOCT	Kolluru et al. [41]	DT	Accuracy	96% ± 0.01%	Under 4 seconds when run on a standard 12-core CPU
	Lee et al. [43]	CNN	Sensitivity/specificity	85.1%/94.2%	0.27 seconds of each image
	Xu et al. [44]	CNN	Accuracy	76.39%	—
MRI	Benedikt et al. [45]	Decision forest	Accuracy	91.8%	—
	Baessler et al. [46]	DL	AUC	0.92	—
Functional diagnosis of CHD	Coenen et al. [55]	ML	—	—	—
	Doeberitz et al. [56]	ML	—	—	—
	Kishi et al. [59]	DL	—	—	59.4 ± 16.0 minutes of average analysis time
	Doeperitz et al. [60]	DL	Accuracy	92%	—
	Yu et al. [66]	DL	Accuracy	90.5%	Median analysis time is 102 seconds
